The article "Accuracy and reproducibility of mouse cortical bone microporosity as quantified by desktop microcomputed tomography" was published in 2017. Journal: PLoS One.

# Accuracy and reproducibility of mouse cortical bone microporosity as quantified by desktop microcomputed tomography

**DOI:** 10.1371/journal.pone.0182996

**Published:** 2017-08-10

**Authors:** Haniyeh Hemmatian, Michaël R. Laurent, Samaneh Ghazanfari, Dirk Vanderschueren, Astrid D. Bakker, Jenneke Klein-Nulend, G. Harry van Lenthe

**Affiliations:** 1 Biomechanics Section, Department of Mechanical Engineering, KU Leuven, Leuven, Belgium; 2 Department of Oral Cell Biology, Academic Centre for Dentistry Amsterdam (ACTA), University of Amsterdam and Vrije Universiteit Amsterdam, Amsterdam Movement Sciences, Amsterdam, The Netherlands; 3 Laboratory of Molecular Endocrinology, Department of Cellular and Molecular Medicine, KU Leuven, Leuven, Belgium; 4 Gerontology and Geriatrics, Department of Clinical and Experimental Medicine, KU Leuven, Leuven, Belgium; 5 Aachen-Maastricht Institute for Biobased Materials, Department of Humanities and Sciences, Maastricht University, Geleen, The Netherlands; 6 Clinical and Experimental Endocrinology, Department of Clinical and Experimental Medicine, KU Leuven, Leuven, Belgium; University of Notre Dame, UNITED STATES

## Abstract

Bone's microporosity plays important roles in bone biology and bone mechanical quality. In this study, we explored the accuracy and reproducibility of nondestructive desktop μCT for 3D visualization and subsequent morphometric analysis of mouse cortical bone microporosity including the vascular canal network and osteocyte lacunae. The accuracy of measurements was evaluated in five murine fibula using confocal laser scanning microscopy (CLSM) in conjunction with Fluorescein isothiocyanate (FITC) staining as the reference method. The reproducibility of μCT-derived cortical bone microstructural indices was examined in 10 fibulae of C57Bl/6J male mice at a nominal resolution of 700 nanometer. Three repeated measurements were made on different days. An excellent correlation between μCT and CLSM was observed for both mean lacuna volume (r = 0.98, p = 0.002) and for mean lacuna orientation (r = 0.93, p = 0.02). Whereas the two techniques showed no significant differences for these parameters, the mean lacuna sphericity acquired from μCT was significantly higher than CLSM (p = 0.01). Reproducibility was high, with precision errors (PE) of 1.57–4.69% for lacuna parameters, and of 1.01–9.45% for vascular canal parameters. Intraclass correlation coefficient (ICC) showed a high reliability of the measurements, ranging from 0.998–1.000 for cortical parameters, 0.973–0.999 for vascular canal parameters and 0.755–0.991 for lacuna parameters. In conclusion, desktop μCT is a valuable tool to quantify the 3D characteristics of bone vascular canals as well as lacunae which can be applied to intact murine bones with high accuracy and reproducibility. Thus, μCT might be an important tool to improve our understanding of the physiological and biomechanical significance of these cannular and lacunar structure in cortical bone.

The article "Accuracy and reproducibility of mouse cortical bone microporosity as quantified by desktop microcomputed tomography" was published in 2017. Journal: PLoS One.

## Introduction

Osteoporosis is a systemic skeletal disease characterized by decreased bone mass as well as deterioration of bone microarchitecture, leading to reduced bone strength and increased risk of fragility fractures [1]. As bone strength does not only depend on bone geometry, but is also influenced by intracortical porosity, improving our understanding of bone microstructure is of great importance to predict mechanical bone properties which in turn are directly related to many metabolic bone diseases [2–6].

Cortical bone is a living dynamic tissue that has a hierarchically organized microstructure which is able to repair and adapt itself dynamically to mechanical and endocrine signals throughout life. Cortical bone morphology is an important determinant of mechanical properties of bone such as stiffness and strength [7]. Cortical bone has an intricate microstructural porosity which, though making up only a few volume percent, is essential in maintaining bone’s adaptive response. The vascular canal network is a major component of the cortical bone microporosity which is altered by remodeling [8] and enables fluid flow throughout the cortex [9,10]. Osteocyte lacunae, which can be considered small micropores encapsulated by bone, make up the second component of bone’s microporosity. Osteocytes, one of the three major bone cell types, reside in these lacunae. These cells are crucial for bone modeling and remodeling since they are considered as mechanosensors in bone [11,12]. From a mechanical point of view, the osteocyte lacunae have been hypothesized to act as stress risers [13], hence, they can have a direct effect on bone fracture behavior. Remodeling-related changes in the structure of bone microporosity affect bone strength and are connected to the functional bone adaptation and disease states such as osteoporosis [14]. Therefore, in order to enhance current physiological understanding on the role the cannular and osteocyte lacunar structure play in bone modeling and remodeling, there is a strong need for a quantitative assessment of bone structure at the submicron level.

Several techniques have been introduced to visualize and quantify bone microstructure. Although quantitative histological and microscopic imaging techniques such as light microscopy, scanning electron microscopy or transmission electron microscopy have provided unique data on bone tissue dynamics [15,16], they cannot provide a complete visualization of bone microstructure as they are based on a few two-dimensional (2D) sections. Additionally, these techniques are destructive and morphological arrangement of the tissue might be influenced by the fixation and sectioning procedures [10,17]. The development of confocal laser scanning microscopy (CLSM) allows to obtain 3D visualization of bone microstructure [16,18,19], but it is limited in the depth of penetration in hard tissue, and the data acquisition and quantification is a time-consuming process [18]. Other 3D recent techniques that are less commonly used are ptychographic X-ray computed tomography (CT) [20], transmission X-ray microscopy CT, transmission electron microscopy CT [21], and serial focused ion beam/scanning electron microscopy (FIB/SEM) [22]. Although these techniques provide 3D representations of bone microstructure at high spatial resolution, they are limited by a small field of view and long acquisition time. Additionally, serial FIB/SEM is a destructive technique and requires extensive sample preparation. In contrast, micro-computed tomography (μCT) is a nondestructive and three-dimensional methodology for characterization of biological tissues. The main advantage of μCT is providing nondestructive quantitative data without preparation of the sample. Afterwards, the sample can still be processed for (dynamic) histomorphometry or immunohistochemistry. Conventional μCT is commonly used in translational bone research to examine cortical and trabecular bone microarchitecture in preclinical rodent models, typically operating around 5–10 μm resolution. Synchrotron radiation-based μCT (SR-μCT) is considered the gold standard when evaluating osteocyte lacunar-canalicular network and their three-dimensional (3D) distribution [15,23–30]. Yet, it comes with a limited field of view and requires dedicated and expensive infrastructure. 3D morphometric properties of the osteocyte lacunar system and distribution have been reported from SR-μCT in human femoral cortical bone [25,26,29]. Cortical osteocyte lacunar density and volume have also been studied in unloaded growing rats based on SR-μCT [30]. Recently, the differences in lacunar geometric properties between lamellar and central bone in rat cortical bone were reported using SR-μCT [27]. Recent developments in desktop μCT systems now allow achieving submicron resolution and has been used to visualize osteocyte lacunae in bone [31–33] and could potentially form an alternative to SR-μCT. Yet, compared to SR-μCT, desktop μCT has lower image quality due to beam hardening and lower signal to noise ratio. Thus, the aim of this study was to visualize and quantify mouse cortical bone microporosity using a desktop μCT system and to evaluate the accuracy and reproducibility of μCT derived mouse cortical bone microstructural parameters.

The article "Accuracy and reproducibility of mouse cortical bone microporosity as quantified by desktop microcomputed tomography" was published in 2017. Journal: PLoS One.

## Materials and methods

### Specimens

For the accuracy study 5 fibulae were used. Three fibulae were extracted from three 5-month-old female C57BL/6JRccHsd mice (21.5 ± 1.3 g) and two fibulae were obtained from two 23-month-old female C57BL/6 mice (28.6 ± 1.9 g). Mice were purchased from Harlan (Horst, The Netherlands). Ethical approval for animal procedures was given by the Animal Ethics Committee of KU Leuven (P075/2015).

The reproducibility study was performed using 10 fibulae which were extracted from 16-week-old male C57BL/6J mice (29 ± 1 g, purchased from Charles Rivers Laboratories). Mice used in the reproducibility study had been used in a non-related study ethically approved by the Animal Ethics Committee of KU Leuven (P143/2011) [34].

All mice were group housed in conventional conditions: 12-hour light, 12-hour dark cycle, standard diet (1% calcium, 0.76% phosphate), and water ad libitum in standard cages as reported previously [34]. Animals were bred and used in accordance with current Belgian national regulations for Animal Welfare and the 2010/63/EU directive. Mice were euthanized by cardiac puncture following deep anesthesia with i.p. pentobarbital (Nembutal, Ceva, Belgium; 100 mg/kg diluted 1:10 in PBS).

### MicroCT imaging

Each fibula was positioned in a custom fixture filled with PBS and scanned using a SkyScan 1172 (Bruker, Kontich, Belgium) μCT scanner. The scan area started at 50% of the whole fibula length (calculated from the growth plate at the proximal part) minus 0.7 mm. The sample was rotated over 180° at a rotation step of 0.2°. The X-ray settings were standardized to 80 kV and 124 μA with an exposure time of 4123 ms. Four times frame averaging was used. The total scan time for one sample was approximately 6 h. One scan produced 2000 contiguous slices with a nominal resolution of 0.7 μm, resulting in a stack height of 1.4 mm. Each slice contained 4000 x 4000 pixels. The scanning parameters at this resolution were selected to enhance the signal-to-noise ratio and the image contrast. The X-ray projections were reconstructed using a modified back-projection [35] reconstruction algorithm (NRecon 1.6.4.6 software-SkyScan) to create cross-sectional images. Reconstruction parameters included ring artifact reduction (RAR = 15), beam hardening correction (BHC = 20%), and misalignment correction. Additionally, a smoothing filter with a Gaussian window kernel (2 pixels) was used to optimize the images.

The article "Accuracy and reproducibility of mouse cortical bone microporosity as quantified by desktop microcomputed tomography" was published in 2017. Journal: PLoS One.

#### MicroCT image processing

A histogram-based global thresholding method was applied to the reconstructed bone to segment the mineralized tissue and nonmineralized structures. Small elements (noise) outside of the cortical bone were removed using the sweep operation in CTAn software (v.1.14.4.1, SkyScan) which removed all but the largest object. Then, intracortical porosity comprising lacunae and vascular canals was segmented by inverting the image and using the 3D despeckled filter in CTAn. The objects less than 100 μm^3^ were considered to be noise (Fig 1A), elements with a volume in the range between 100 and 2000 μm^3^ were assumed to be osteocyte lacunae (Fig 1B), and the objects greater than 2000 μm^3^ were considered to be vascular canals (Fig 1C). These volume limits were used in previous synchrotron-based studies [25,36] and were based on the confocal microscopy measurements indicating a size between 28–1713 μm^3^ for each osteocyte [37]. Note that canaliculi were not segmented since their size was below the scan resolution used in this study. 3D renderings of the lacunae and vascular canal network (Fig 2) were created using CTVox software (v.3.3.0, SkyScan).

**Fig 1:** Volume filtering of μCT-derived cortical bone microporosity comprising lacunae and vascular canals. Pores were classified as (A) noise (<100 μm^3^); (B) lacunae (100–2000 μm^3^); (C) vascular canals (>2000 μm^3^). Scale bar = 100 μm.

**Fig 2:** 3D rendering of μCT-derived cortical bone microporosity including osteocyte lacunae and vascular canal network of mouse fibula. Yellow: osteocyte lacunae; red: vascular canal network. Scale bar = 100 μm.

#### MicroCT 3D morphometric evaluation

We derived morphometric measures for the bone [38] using CTAn, including total tissue volume (TV) (including medullary canal and the cortical bone tissue), cortical total volume (Ct.TV) (comprising the cortical bone volume together with lacunae and vascular canal network), cortical bone volume (Ct.BV) (excluding porosities), cortical bone volume density (Ct.BV/TV), cortical thickness (Ct.Th), polar moment of inertia (J), and mean periosteal perimeter (Ps.Pm) at macro-level. The vascular canal network on the micro-level was quantitatively determined by the following parameters: total canal volume (Ca.V), canal volume density (Ca.V/Ct.TV), canal number (Ca.N), canal number density (Ca.N/Ct.TV), mean canal orientation (Ca.θ), mean canal length (Ca.Le), and mean canal diameter (Ca.Dm), where the canal diameter was calculated using the “sphere fitting” method developed by Hildebrand and Rüegsegger [39] and canal length was calculated as mean canal volume (Ca.V/N.Ca) divided by the canal cross section area (π·(Ca.Dm/2)^2^). Similarly, the lacunar network was determined by quantifying total lacuna volume (Lc.V), lacuna number (N.Lc), lacuna volume density (Lc.V/Ct.TV), lacuna number density (N.Lc/Ct.TV), mean lacuna volume (<Lc.V> = Lc.V/N.Lc), mean lacuna orientation (Lc.θ), and mean lacuna sphericity (Lc.Sph). The lacuna number density was quantified as the number of 3D objects per unit volume. The lacuna sphericity was calculated as the ratio of the surface area of a sphere with the same volume as the given lacuna to the lacuna surface area. The lacuna and canal orientation were calculated from the fibula longitudinal axis.

The article "Accuracy and reproducibility of mouse cortical bone microporosity as quantified by desktop microcomputed tomography" was published in 2017. Journal: PLoS One.

### Confocal microscopy imaging and analyses

2 mm of the middle part of each bone was cut and dehydrated in ascending graded ethanol. Subsequently, the samples were stained with fluorescein isothiocyanate isomer I (FITC) diluted in absolute EtOH at a concentration of 1% for 24 h, similar to the method described by Ciani et al.[40] The samples were then washed for 1 h in 100% ethanol and mounted on coverslips using Vectashield mounting media (Vector Laboratories, Burlingame, CA).

The bone samples were imaged (Fig 3A) using a confocal microscope (Leica SP8, Germany) with the following parameters: 40× oil immersion lens, 1.25 numerical aperture, laser wavelength excitation of 488 nm, pinhole set at 1, 1024 × 1024 resolution with a pixel size of 0.4 μm, and laser intensity set at 10% of the full power. The distance between two adjacent optical slices was set to 0.7 μm.

**Fig 3:** Osteocyte lacunae visualized by using confocal laser scanning microscopy (CLSM). (A) a z-projection of confocal imaging of osteocyte lacunae in the mouse cortical bone stained with FITC (fluorescein isothiocyanate isomer I, Sigma). (B) CLSM-based 3D renderings of osteocyte lacunae. The dark green lacunae correspond to in-plane lacunae shown in the microscopy image (A). Scale bar = 20 μm.

Using CTAn software the osteocyte lacunar network were segmented from CLSM images. After thresholding, an erosion operation followed by a dilation operation was used in CTAn to remove the stained canaliculae. 3D renderings of the osteocyte lacunar network were created by Mimics software (Fig 3B). Subsequently, quantitative histomorphometric indices of osteocyte lacunar network including mean lacuna volume (<Lc.V>), mean lacuna orientation (Lc.θ), and mean lacuna sphericity (Lc.Sph) were calculated using CTAn software in the regions which were well stained.

### Accuracy study

To quantify the accuracy, after fixing the bones overnight in 2% PBS-buffered paraformaldehyde at 4°C, 1.4 mm of the middle part of each fibula was scanned at a nominal resolution of 0.7 μm using desktop μCT. Following μCT scanning, 2 mm of the middle part of each bone was cut and stained with FITC. The samples were then imaged using CLSM. Since the imaging depth was limited to approximately 100 μm, the bone samples were visualized from both the lateral and medial sides. To assess the accuracy, the lacunae parameters acquired from CLSM were compared with that from μCT measured in the corresponding volumes of interest.

The article "Accuracy and reproducibility of mouse cortical bone microporosity as quantified by desktop microcomputed tomography" was published in 2017. Journal: PLoS One.

### Reproducibility study

To quantify the reproducibility, samples were scanned three times using μCT and after each scan the samples were repositioned. After reconstruction and segmentation, 800 slices of the common regions in three scans were selected and analyzed. To find overlapping regions between scans a 3D rigid registration method was applied, where the second and the third images were registered to the first one (reference image). The overlap between the masks of three scans represents the largest common volume.

### Statistics

The accuracy of μCT was assessed by computing Pearson correlation coefficients and 95% agreement limits in accordance with Bland-Altman analysis [41]. A paired t test was performed to evaluate whether the differences between μCT and CLSM were significant. These statistical analyses were performed using GraphPad Prism version 6.0 for Windows (GraphPad Software, La Jolla, CA, USA). For the accuracy study, no power calculation was performed to determine sample size because of lack of data at the start of the study.

For the reproducibility study, 3 repeated measurements on 10 samples, hence, providing 20 degrees of freedom, indicates that the upper confidence limit of the precision error is 40% higher than the mean precision error [42]. Reproducibility was determined by calculating precision error (PE_%CV_) and intraclass correlation coefficient (ICC). To evaluate the reproducibility of μCT derived cortical bone microstructural parameters, PEs were defined as the root mean square coefficient of variance. For each parameter we computed PEs both in absolute values (PE_SD_) and as coefficient of variation (PE_%CV_) of repeated measurements on a percentage basis as described previously in detail by Gluer et al. [42]:

$$PE_{SD}=\sqrt{\sum_{j=1}^{m}\frac{SD_{j}^{2}}{m}}$$ (1)

$$PE_{\%CV}=\sqrt{\sum_{j=1}^{m}\frac{\%CV_{j}^{2}}{m}}$$ (2)

Where m is the number of subjects, SD is the standard deviation of n repeated measurements on a given subject j, and the coefficient of variation was calculated as follows: $\%CV_{j}=SD_{j}/{\bar{x}}_{j}.100\%$. The result of the ith measurement for subject j is *x*_*ij*_ and ${\bar{x}}_{j}$ is the mean of all *x*_*ij*_ for subject j. For each of the PE_%CV_, a confidence interval was also calculated to determine the accuracy of PEs.

The article "Accuracy and reproducibility of mouse cortical bone microporosity as quantified by desktop microcomputed tomography" was published in 2017. Journal: PLoS One.

We quantified the intraclass correlation coefficients (ICC) as introduced by Shrout and Fleiss [43]. ICC is defined as the ratio of the intrasubject variance over the population variance. The values vary between 0 and 1 where 1 represents perfect reproducibility. The appropriate form of ICC for this study corresponds to the two-way mixed model ICC (3,1) as described by Shrout and Fleiss [43] and has been calculated as follows:

$$ICC=\frac{F_{0}-1}{F_{0}+\left(n-1\right)}$$ (3)

*F*_0_ is the ratio of between-subject mean squares and the residual within-subject mean squares and n is the number of repetitions. In this model, the subjects are treated as random effects. However, the number of repetitions are considered as fixed effects where they are the only ones of interest. Statistical analyses were performed using Excel 2010 (Microsoft, Redmond, OR, USA) and Matlab (The Mathworks, Inc., Natick, MA, USA).

## Results

Using a high-resolution desktop μCT system, the microposity of mouse cortical bone was visualized and quantified. The segmentation process resulted in separation of bone and microporosity (see Materials and methods). Pores were classified as lacunae and vascular canals using volume filtering (Fig 1). 3D rendering of cortical bone microporosity of the fibula indicated that the current method was able to reveal different structures of cortical bone microporosity comprising lacunae and vascular canal network (Fig 2).

The comparison between μCT-derived morphometric parameters and CLSM showed a good agreement between the two techniques (Table 1, Fig 4). The highest correlation between μCT and CLSM was found for mean lacuna volume (r = 0.98, p = 0.002). Based on Bland-Altman analysis (Fig 4D), the mean differences (μCT minus CLSM) in Lc.V was 7.49 μm^3^. The lower and upper limits of agreement between the two methods were -23.70 μm^3^ and 38.69 μm^3^, respectively. The mean lacuna volume derived from μCT was 235.9 ± 39.83 μm^3^ and it was not significantly (p = 0.35) different from that of CLSM (228.4 ± 24.77 μm^3^). The correlation coefficient between μCT and CLSM for <Lc.Ɵ> was 0.93 (p-value = 0.02). Using Bland-Altman analysis (Fig 4E), the mean differences (μCT minus CLSM) in <Lc.Ɵ> was -0.84° (95% limits of agreement -2.80 to 1.11°). There was a negative relationship between μCT-derived and CLSM-based sphericity of lacuna (r = -0.37, p = 0.54). The mean value of lacuna sphericity was significantly (p = 0.01) lower from CLSM (0.48 ± 0.03) than from μCT (0.59 ± 0.02). Bland–Altman plot shows agreement between the μCT-derived and CLSM-based measurement of Lc.Sph (Fig 4F).

The article "Accuracy and reproducibility of mouse cortical bone microporosity as quantified by desktop microcomputed tomography" was published in 2017. Journal: PLoS One.

**Fig 4:** Accuracy analyses of μCT-based osteocyte lacuna parameters vs. those obtained from confocal laser scanning microscopy. Frequency distribution of osteocyte lacuna volume (4A), orientation (4B) and sphericity (4C); Bland-Altman analyses of mean lacuna volume (4D), orientation (4E) and sphericity (4F). The horizontal dashed lines show the 95% limits of agreement and the horizontal solid line shows the mean difference between the two methods. Correlation between mean osteocyte lacuna volume (4G), orientation (4H), and sphericity (4I). μCT = micro-computed tomography; CLSM = confocal laser scanning microscopy; N.Lc = lacuna number; <Lc.V> = mean lacuna volume; Lc.Sph = mean lacuna sphericity; Lc.θ = mean lacuna orientation.

**Table 1:** Accuracy of μCT-derived lacuna parameters.

	Accuracy (μCT vs CLSM)		
Lacuna parameters	Pearson Correlation (r, p)	Paired t test (p)	Bland-Altman Bias, (95% limits of agreement)
**<Lc.V>, μm**^**3**^	0.98, 0.002	0.35	7.49, (-23.70–38.69)
**Lc.θ, °**	0.93, 0.02	0.13	-0.84, (-2.80–1.11)
**Lc.Sph**	-0.37, 0.54	0.01	0.11, (0.02–0.21)

μCT = micro-computed tomography; CLSM = confocal laser scanning microscopy; r = Pearson correlation coefficient; p = p-value; <Lc.V> = mean lacuna volume; Lc.θ = mean lacuna orientation; Lc.Sph = mean lacuna sphericity.

Average lacuna porosity (Lc.V/TV) and vascular canal porosity (Ca.V/TV), measured using μCT were 1.52% and 0.46% respectively. The PE_%CV_ for cortical bone parameters ranged from 0.12% (Ct.BV/TV) to 0.81% (J), for the lacuna parameters from 1.57% (N.Lc) to 4.69% (Lc.Sph) and for vascular canal parameters from 1.01% (Ca.θ) to 9.45% (Ca.Le) (Table 2). The reproducibility for cortical bone parameters with an average PE of 0.44% were observed to be highest, followed by lacuna parameters (average PE = 3.19%) and vascular canal parameters (average PE = 5.05%).

**Table 2:** Morphometric parameters, precision errors, and confidence intervals for repeated analysis used in this study.

Morphometric parameters		Mean	PE_SD_	PE_%CV_	0.95% CI PE_%CV_
**Cortical bone parameters**	TV (mm^3^)	0.087	0.0003	0.36%	0.33–0.52%
	Ct.TV (mm^3^)	0.068	0.0005	0.73%	0.67–1.06%
	Ct.BV (mm^3^)	0.066	0.0002	0.39%	0.36–0.57%
	Ct.BV/TV (%)	77.23	0.0915	0.12%	0.08–0.13%
	Ct.Th (μm)	139.59	0.4846	0.35%	0.32–0.50%
	J (mm^4^)	0.0040	3x10^-5^	0.81%	0.74–1.17%
	Tt.Ar (mm^2^)	0.15	0.0007	0.47%	0.43–0.68%
	B.Ar (mm^2^)	0.12	0.0005	0.42%	0.38–0.61%
	Ps.Pm (mm)	1.60	0.005	0.29%	0.27–0.43%
**Vascular canal parameters**	Ca.V (mm^3^)	0.00031	1x10^-5^	3.53%	3.24–5.10%
	Ca.V/Ct.TV (%)	0.46	0.016	3.52%	3.23–4.67%
	Ca.V/N.Ca (mm^3^)	1.5x10^-5^	9x10^-7^	6.04%	5.54–8.73%
	N.Ca	20.57	1.3784	6.70%	6.14–9.68%
	N.Ca/Ct.TV (mm^-3^)	302.69	20.706	6.84%	6.27–9.88%
	Ca.θ (°)	45.80	0.4643	1.01%	0.93–1.46%
	Ca.Dm (μm)	9.1	0.3	3.33%	3.05–4.81%
	Ca.Le (mm)	0.26	0.0250	9.45%	8.66–13.65%
**Lacuna parameters**	N.Lc	2875	45.049	1.57%	1.44–2.26%
	Lc.V (mm^3^)	0.00104	3x10^-5^	3.12%	2.86–4.52%
	Lc.V/Ct.TV (%)	1.52	0.0471	3.09%	2.83–4.46%
	N.Lc/Ct.TV (mm^-3^)	42218.2	831.85	1.97%	1.81–2.84%
	Lc.V/N.Lc (mm^3^)	3.6x10^-7^	1x10^-8^	3.44%	3.15–4.96%
	Lc.θ (°)	7.43	0.2077	2.80%	2.56–4.04%
	Lc.Sph	0.60	0.0283	4.69%	4.30–6.77%

Mean = the mean of morphometric parameters; PE_SD_ = precision errors expressed in absolute values; PE_%CV_ = precision errors expressed as coefficient of variation of repeated measurements; 0.95% CI PE_%CV_ = 95% confidence interval for PE_%CV_; TV = total tissue volume; Ct.TV = cortical total volume (comprising the cortical bone volume together with lacunae and vascular canal network); Ct.BV = cortical bone volume; Ct.BV/TV = cortical bone volume density; Ct.Th = cortical thickness; J = polar moment of inertia; Tt.Ar = total cross-sectional area inside the periosteal envelope; B.Ar = Cortical bone area; Ps.Pm = periosteal perimeter; Ca.V = total canal volume; Ca.V/Ct.TV = canal volume density; Ca.N = canal number; Ca.N/Ct.TV = canal number density; Ca.θ = mean canal orientation; Ca.Le = mean canal length; Ca.Dm = mean canal diameter; Ca.Le = canal length; N.Lc = lacuna number; Lc.V = total lacuna volume; Lc.V/Ct.TV = lacuna volume density; N.Lc/Ct.TV = lacuna number density; Lc.V/N.Lc = mean lacuna volume; Lc.Sph = mean lacuna sphericity; Lc.θ = mean lacuna orientation.

The article "Accuracy and reproducibility of mouse cortical bone microporosity as quantified by desktop microcomputed tomography" was published in 2017. Journal: PLoS One.

ICC revealed a very high reliability of the measurements, showing that the variances within repeated measurements are smaller than the population variances. The ICC for cortical bone parameters ranged from 0.998 to 1.000, for vascular canal parameter from 0.973 (Ca.Le) to 0.999 (Ca.θ) and for lacuna parameters from 0.755 (Lc.Sph) to 0.991 (N.Lc). The ICC values and their corresponding 95% CIs are presented in Table 3.

**Table 3:** Intraclass correlation coefficients and confidence intervals for repeated analysis.

Morphometric parameters		ICC	95% CI ICC
**Cortical bone parameters**	TV (mm^3^)	1.000	1.000–1.000
	Ct.TV (mm^3^)	0.998	0.992–1.000
	Ct.BV (mm^3^)	0.999	0.998–1.000
	Ct.BV/TV (%)	1.000	1.000–1.000
	Ct.Th (μm)	1.000	0.999–1.000
	J (mm^4^)	1.000	0.999–1.000
	Tt.Ar (mm^2^)	1.000	0.999–1.000
	B.Ar (mm^2^)	0.999	0.998–1.000
	Ps.Pm (mm)	1.000	0.999–1.000
**Vascular canal parameters**	Ca.V (mm^3^)	0.994	0.982–0.998
	Ca.V/Ct.TV (%)	0.990	0.970–0.997
	Ca.V/N.Ca (mm^3^)	0.997	0.888–0.994
	N.Ca	0.974	0.915–0.993
	N.Ca/Ct.TV (mm^-3^)	0.974	0.917–0.993
	Ca.θ (°)	0.999	0.998–1.000
	Ca.Dm (μm)	0.993	0.979–0.998
	Ca.Le (mm)	0.973	0.903–0.993
**Lacuna parameters**	N.Lc	0.991	0.974–0.998
	Lc.V (mm^3^)	0.973	0.922–0.993
	Lc.V/Ct.TV (%)	0.974	0.926–0.993
	N.Lc/Ct.TV (mm^-3^)	0.953	0.867–0.987
	Lc.V/N.Lc (mm^3^)	0.915	0.761–0.977
	Lc.θ (°)	0.918	0.769–0.978
	Lc.Sph	0.755	0.292–0.933

ICC = intraclass correlation coefficient; 95% CI ICC = 95% confidence interval for ICC; TV = total tissue volume; Ct.TV = cortical total volume (comprising the cortical bone volume together with lacunae and vascular canal network); Ct.BV = cortical bone volume; Ct.BV/TV = cortical bone volume density; Ct.Th = cortical thickness; J = polar moment of inertia; Tt.Ar = total cross-sectional area inside the periosteal envelope; B.Ar = Cortical bone area; Ps.Pm = periosteal perimeter; Ca.V = total canal volume; Ca.V/Ct.TV = canal volume density; Ca.N = canal number; Ca.N/Ct.TV = canal number density; Ca.θ = mean canal orientation; Ca.Le = mean canal length; Ca.Dm = mean canal diameter; Ca.Le = canal length; N.Lc = lacuna number; Lc.V = total lacuna volume; Lc.V/ Ct.TV = lacuna volume density; N.Lc/Ct.TV = lacuna number density; Lc.V/N.Lc = mean lacuna volume; Lc.Sph = mean lacuna sphericity; Lc.θ = mean lacuna orientation.

The article "Accuracy and reproducibility of mouse cortical bone microporosity as quantified by desktop microcomputed tomography" was published in 2017. Journal: PLoS One.

## Discussion

In the current study we visualized and quantified the 3D microporosity of cortical bone using desktop μCT. By evaluating the accuracy and reproducibility of μCT measurements in the fibulae of mice, we found that μCT has high accuracy and precision, such that it can be used as a reliable tool for nondestructive measurements of microstructural bone parameters.

The advantage of using murine fibulae was that their small size facilitated analysis by μCT since a single field of view (2 mm) encompassed the entire bone’s cross section; hence no cutting nor preparation was required. Furthermore, the fibula is a load-bearing bone that adapts to mechanical loading in a similar way as the tibia. Several groups have successfully used fibulae to study skeletal mechanobiology [31,34,44].

To our knowledge this paper is the first study using desktop μCT to evaluate the reproducibility of μCT measurement of 3D characteristics of bone vascular canals and the lacunae in entire murine bones. Our accuracy analysis showed a strong correlation between μCT and CLSM demonstrating that murine cortical bone microporosity parameters obtained by the two techniques are similar. μCT revealed a high correlation with CLSM for mean lacuna volume as well as mean lacuna orientation. The accuracy values and comparison between the histograms for lacuna volume and orientation from μCT were in a close agreement with those from CLSM. Despite that the precision error obtained for lacuna sphericity was low (PE = 4.69%), the results of accuracy analysis showed a significant bias of 0.11 indicating that the sphericity was overestimated by μCT. The source of this overestimation is unclear, but could be related to image processing to segment the osteocyte lacunae.

The article "Accuracy and reproducibility of mouse cortical bone microporosity as quantified by desktop microcomputed tomography" was published in 2017. Journal: PLoS One.

The absolute values we obtained for desktop μCT-based analyses on the canals and osteocyte lacunae (Table 2) were in agreement with those found in SRμCT-based analyses. More specifically, the 1.52% average lacunar porosity we found is in line with the reported 1.2%-1.4% using 0.7-micron resolution in mice [23], and the 1.5% using 0.75-micron resolution in rats [36]. The average osteocyte lacuna number density we found (42×10^3^ lacunae per mm^3^) is also similar to the published SR-μCT measurements in mice and rats (49.0×10^3^ to 66.0×10^3^ lacunae per mm^3^) [23,36]. The mean lacuna volume (360 μm^3^) we found in mouse fibula is in accordance with values reported by others [23,31,45]. A mean osteocyte lacuna volume of 200 μm^3^ has been measured using SR μCT in the femoral mid-diaphysis of mice with low bone volume, and a mean osteocyte lacuna volume of 269 μm^3^ in mice with a high bone volume [23]. Osteocyte lacuna volumes of 575 μm^3^ and 366 μm^3^ were measured using nanoCT in mouse fibula and calvaria, respectively [31]. High resolution desktop μCT is capable of achieving osteocyte lacuna sphericity as well as lacuna and canal orientation quantitatively and qualitatively. Using our 3D models of osteocyte lacuna we observed that most lacuna are ellipsoidal shaped with an average sphericity of 0.60, and oriented with the longest osteocyte lacunar axis parallel to the longitudinal direction of the fibula (mean Lc.θ = 7.43°). These finding are in agreement with those by Vatsa et al. [31] in mouse fibula, who demonstrated that osteocyte lacunae in fibulae were more elongated than those in calvarial bone. In addition, the results of current research are also in agreement with the values found recently by Palacio-Mancheno et al. [32] who demonstrated that the nominal resolution should be 1 μm or better to allow quantification of osteocyte lacunar pores and that a nominal resolution of 1 to 2 μm is appropriate to quantify intracortical vascular pores.

A weakness of the CLSM technique is that not all the osteocyte lacuna were stained. Since bone is a non-homogenous material in density and the osteocyte lacuna are deeply embedded in the bone matrix, the staining of all lacunae is hindered by probe diffusion and uneven staining which results in an underestimation of lacuna density. Therefore, the accuracy of osteocyte lacuna number and volume density could not be validated versus CLSM. Furthermore, the accuracy analysis has not been done for the vascular canal parameters. Since the imaging depth was limited to approximately 100 μm (60 μm in practice), the bone samples were visualized from both the lateral and medial sides. In these small regions of interest there are not enough canals to assess the accuracy. The validation of μCT in characterizing cortical bone porosity at the level of vascular canals has been previously reported in the literature [17,46–49]. A good correlation (R^2^ = 0.97) was found for cortical porosity, Haversian canal diameter and canal separation as measured by μCT with a spatial resolution of 8 μm and 2D histological sections as a reference method [46]. μCT measurement of human cortical bone porosity (Volkmann and Havers canals) was also validated against scanning electron microscopy (SEM) measurements. Porosity obtained by μCT with a spatial resolution of 8 μm was correlated with porosity measured by SEM (r = 0.91, p<0.05) [49].

The article "Accuracy and reproducibility of mouse cortical bone microporosity as quantified by desktop microcomputed tomography" was published in 2017. Journal: PLoS One.

Cortical bone parameters showed lowest (best) PEs values, followed by lacuna parameters and vascular canal indices. Since μCT imaging is based on X-ray attenuation, and since the bone tissue forms the largest constituent of the samples, it is not surprising that the PEs of cortical bone parameters are better than those of the vascular canal and lacuna parameters. The precision errors of canal parameters were higher than those of lacuna parameters. This is because only a few canals were present in the samples, while at the same time they experienced relatively large variations; this is in contrast to the lacunae which were much more abundant and saw less variation. The highest (worst) precision error was found for canal length. We hypothesize that the image resolution does not suffice to precisely identify all connections between smaller canals such that canals can appear separated whereas in reality they form one entity. Furthermore, as the canal length was calculated as the mean canal volume (Ca.V/N.Ca) divided by the canal cross section area (π·(Ca.Dm/2)^2^), its reproducibility is affected by the reproducibility of Ca.V, N.Ca, and Ca.Dm. Yet, ICC values were high, from which can be concluded that the within-repeated measurements variances were much smaller in comparison with the population variances, such that it is possible to make a clear distinction between different specimens.

ICC ranged from 0.755 to 1.000, hence, showed a very high reliability of the measurements, indicating that the variances within repeated measurements are very small in comparison with the population variances. The ICC values of the lacuna parameters were lower as compared to the cortical bone and vascular canal parameters, indicating that there are large number of lacunae with less variation in a small volume of interest. The high ICC values show that the analysis procedure presented in this study is a reliable technique to assess bone microstructural indices in the mouse fibula.

The article "Accuracy and reproducibility of mouse cortical bone microporosity as quantified by desktop microcomputed tomography" was published in 2017. Journal: PLoS One.

In summary, we achieved non-destructive 3D visualization of cortical microporosity in a mouse appendicular long bone. By using a high-resolution desktop μCT system and quantification software, we were able to (i) visualize the intracortical porosity in the mouse fibula, (ii) decompose it into the vascular canal network and the osteocyte lacunar system, (iii) quantify their morphometric characteristics, (iv) validate their accuracy and reproducibility. We conclude that desktop μCT, which is more readily available than SR μCT for many investigators, can aid studies on biological influences on microarchitectural properties like vascular canals and lacunae with a high accuracy and precision. Furthermore, it can bring the required data to enhance our understanding of the role of these microarchitectural features in bone modeling and remodeling.

## Supporting information

S1 Dataset Accuracy data. Data used to evaluate accuracy.
(XLSX)

S2 Dataset Reproducibility data. Data used to evaluate reproducibility.
(XLSX)
